# Hyperspectral Image Classification: Potentials, Challenges, and Future Directions

**DOI:** 10.1155/2022/3854635

**Published:** 2022-04-28

**Authors:** Debaleena Datta, Pradeep Kumar Mallick, Akash Kumar Bhoi, Muhammad Fazal Ijaz, Jana Shafi, Jaeyoung Choi

**Affiliations:** ^1^School of Computer Engineering, Kalinga Institute of Industrial Technology, Deemed to be University, Bhubaneswar 751024, India; ^2^KIET Group of Institutions, Delhi-NCR, Ghaziabad-201206, India; ^3^Directorate of Research, Sikkim Manipal University, Gangtok 737102, Sikkim, India; ^4^AB-Tech eResearch (ABTeR), Sambalpur, Burla 768018, India; ^5^Department of Intelligent Mechatronics Engineering, Sejong University, Seoul 05006, Republic of Korea; ^6^Department of Computer Science, College of Arts and Science, Prince Sattam Bin Abdul Aziz University, Wadi Ad-Dawasir 11991, Saudi Arabia; ^7^School of Computing, Gachon University, Seongnam-si 13120, Republic of Korea

## Abstract

Recent imaging science and technology discoveries have considered hyperspectral imagery and remote sensing. The current intelligent technologies, such as support vector machines, sparse representations, active learning, extreme learning machines, transfer learning, and deep learning, are typically based on the learning of the machines. These techniques enrich the processing of such three-dimensional, multiple bands, and high-resolution images with their precision and fidelity. This article presents an extensive survey depicting machine-dependent technologies' contributions and deep learning on landcover classification based on hyperspectral images. The objective of this study is three-fold. First, after reading a large pool of Web of Science (WoS), Scopus, SCI, and SCIE-indexed and SCIE-related articles, we provide a novel approach for review work that is entirely systematic and aids in the inspiration of finding research gaps and developing embedded questions. Second, we emphasize contemporary advances in machine learning (ML) methods for identifying hyperspectral images, with a brief, organized overview and a thorough assessment of the literature involved. Finally, we draw the conclusions to assist researchers in expanding their understanding of the relationship between machine learning and hyperspectral images for future research.

## 1. Introduction

Hyperspectral imagery is one of the most significant discoveries in remote sensing imaging sciences and technological advancements. Hyperspectral imagery (HSI) is the technology that depicts the perfect combination of Geographic Information System (GIS) and remote sensing. Besides, HSI has several advantages such as ecological protection, security, agriculture and horticulture applications, crop specification and monitoring, medical diagnosis, identification, and quantification [1]. RGB images are made up of three dimensions: width, height, and 3 color bands or channels consisting of color information, that is, red, green, and blue. They are stored as a 3D byte array that explicitly holds a color value for each pixel in the image; a combination of RGB intensities put down onto a color plane. However, in contrast, HSI comprises thousands of hypercubes and hence possesses a large resolution and an enormous amount of embedded information of all kinds—spectral, spatial, and temporal. This information enables various applications to detect and characterize land covers, which are most significantly explored [2]. RGB images are captured by digital RGB cameras capable of characterizing objects only based on their shape and color. Moreover, the embedded information is minimal since only three visible bands are available in the human visibility range. The HSI, on the other hand, is captured by specialized airborne hyperspectral sensors placed on artificial satellites, that is, spectrometers. They have a broad range of scenes by acquiring large numbers of consecutive bands, not confined to the visible light spectrum and through a wider spectral band-pass. However, compared to the digital sensor that absorbs light in just three wide channels, a hyperspectral sensor's channel width is much narrower, making the spectral resolution and data volume much higher, resulting in hurdles to store, mine, and manage [3]. Furthermore, processing these data with a massive number of bands imposes many obstacles such as noise-causing image calibration, geometric distortion, noisy labels, and limited or unbalanced labeled training samples [4–6], that is, Hughes phenomenon and dimensionality reduction-related artifacts: overfitting, redundancy, spectral variability, loss of significant features between the channels, etc. [7].

Classifying HSIs is considered to be an intrinsically nonlinear problem [8], and the initial approach by linear-transformation-based statistical techniques such as principle component analytical methods, that is, principal component analysis (PCA) [9] and independent component analysis (ICA) [10]; the discriminant analytical methods, that is, linear [11] and fisher [12]; wavelet transforms [13]; and composite [14], probabilistic [15], and generalized [16] kernel methods, had shown promising outcomes. Still, their focus was limited to spatial information. They emphasized that the feature extractor techniques assisted by some basic random classifiers that lead to complexity in terms of cost, space, and time are not sufficiently accurate. After the success of these traditional methodical techniques assigned for HSI classification, researchers became keenly interested in applying the most recent emerging but not tedious computer-based methods that made the entire process smoother and vicinal to perfection. Study advancements suggest that the last decade can be considered the most escalating era regarding computer-based technologies due to the emergence of machine learning (ML). ML is an algorithmic and powerful tool that resembles the human brain's cognition. It simply represents a complex system by holding abstraction. Hence, it can reduce complexities and peep into the insights of the vast amount of HS data to fetch out the hidden discriminative features, both spectral and spatial [17]. Thus, it overcomes all the stumbling blocks to achieve the desired accuracy in identifying the classes that the objects of the target HSI data belong to. Hence, they act as all-in-one techniques that can serve the purpose without further assistance. Keeping this in mind, we conducted an extensive survey based on the various discriminative machine and deep learning (ML, DL) models for HSI. In most of the literature studies, the HSI datasets that are commonly used for landcover classification are AVIRIS Indian Pines (IP), Kennedy Space Center (KSC), Salinas Valley (SV), and ROSIS-03 University of Pavia (UP), along with less frequently used Pavia Center, Botswana, University of Houston (HU), etc. They are pre-refined and made publicly available on [18] for download and perform operations.

The motivation of our work is divided into three parts. First, a novel methodology is proposed for the review work that is entirely systematic and helps find the inspiration in forming the research gaps and embedded questions after going through a large pool of research articles. Second, this work focuses on the current advancements of ML technologies for classifying HSI, with their brief, methodical description and a detailed review of the literature involved with them. Finally, the inferences are drawn and help the researchers boost knowledge for their future research. The key contributions made to the research field on hyperspectral imagery by our novel effort are as follows:

1. The thorough revision of the analytical and classification work carried out to date on HS imagery by employing ML/DL techniques.
2. Emphasis on the categorized methods explored and practiced so far in an overly frequent manner. Also, it includes a brief interpretation of the most recent technologies and the highlighted hybrid techniques.
3. An open knowledge base that acts as a reservoir of relevant information that is listed out that interprets all research on each mentioned technique in terms of their methodology, convenience and limitations, and future strategies. This illustration might administrate in making a proper choice of objective for further research on the field of HSIs.
4. Explicit idea of the growth of interest in the concerned field that would attract researchers to invest themselves with a coherent, substantial specification (benefaction and drawbacks) of all the methods, individually, that contributes academically to the researchers about their favorable result and the difficulties for a chosen technique.
5. A transitory rendition of the most recent research on HSIs signifies the currently adapted technologies as hot spots. Also, focus on the research areas about the interest that could apply to others, that is, the hybridized methods popular among researchers to address the problem and achieve the desired experimental results.

The rest of the article is arranged as follows: Section 2 briefly explains the constraints faced by the researchers in dealing with HSI; Section 3 represents the methodology for the research along with the motive behind this review; Section 4 describes seven ML techniques, namely, support vector machine (SVM), sparse representation (SR), Markov random field (MRF), extreme learning machine (ELM), active learning (AL), deep learning (DL), and transfer learning (TL); Section 5 shows up the complete summary of the literature review work in the form of answers to the research questions; Section 6 depicts the conclusions; and Section 7 explains the limitations and future work.

## 2. Constraints of HSI Classification

Since their emergence, several difficulties have caused issues in analyzing and performing operations on hyperspectral images. Initially, it suffered from spectroscopy technology due to the bad quality of hyperspectral sensors and poor quality with insufficient data. However, along with the advancement in applied science, things have come to ease, but there are still some well-known nondispersible hitches that need to be overcome. Some of them are stated as follows:

- Lack of high-resolution Earth observation (EO) noiseless images: During the initial stage of the discovery of spectrometers, they were not very efficient. Due to this, noises caused by water vapor, atmospheric pollutants, and other atmospheric perturbations modify the signals coming from the Earth's surface for Earth observations. Several efforts have been made over the last decades to produce high-quality hyperspectral data for Earth observation and develop a wide range of high-performance spectrometers that combines the power of digital imaging, spectroscopy, and extracting numerous embedded spatial-spectral features [19].
- Hindrances in the extraction of features: During data gathering, redundancy across contiguous spectral bands results in the availability of duplicated information, both spatially and spectrally, obstructing the optimal and discriminative retrieval of spatial-spectral characteristics [7].
- The large spatial variability and interclass similarity: The hyperspectral dataset collected contains unusable noisy bands due to mistakes in the acquisition that result in information loss in terms of the unique identity, that is, the spectral signatures and excessive intraclass variability. Furthermore, with poor resolution, each pixel comprises broad spatial regions on the Earth's surface, generating spectral signature mixing, contributing to the enhanced interclass similarity in border regions, thus creating inconsistencies and uncertainties for employed classification algorithms [19].
- Limitation of available training samples and insufficient labeled data: Aerial spectrometers cover significantly smaller areas, so they can only collect a limited number of hyperspectral data. That leads to the restriction of the number of training samples for classification models [20]. In addition, HSIs typically contain classes that correspond to a single scene, and available classification models' learning procedures require labeled data. However, labeling each pixel requires human skill, which is arduous and time-consuming [21].
- Lack of balance among interclass samples: The class imbalance problems, where each class sample has a wide range of occurrences, diminish the usefulness of many existing algorithms in terms of enhancing minority class accuracy without compromising majority class accuracy, which is a difficult task in and of itself [22].
- The higher dimensionality: Due to incorporating more information in multiple channels, such high-band pictures increase estimation errors. The curse of dimensionality is a significant drawback for supervised classification algorithms, as it significantly impacts their performance and accuracy [23].

The possible solutions to the above limitations that also represent the possible operations that are performed to analyze and comprehend the HSIs can be (1) technological advancement to make versatile and robust hardware for the spectrometers to capture the scenes more accurately, (2) spectral unmixing and resolution enhancement for better feature extraction and distinguishing capability of the embedded objects, (3) image compression-restoration and dimensionality reduction for addressing the high-dimensions and lack of data, and (4) use of robust classifiers that are capable of dealing with the above issues as well as promote fast computation ability [7].

These hurdles were very prominent for the methods that classify HSI based on the feature extrication from HSI. After ML/DL came into the scene, the operations on HSI became effortless as explicit feature extraction is not needed, and it has also many advantages such as great dealing with noise and time complexity. However, ML/DL acquires a few drawbacks in specific criteria [19], including parameter-tuning and numerous local minima problems in training procedures and compression [20] overfitting, optimization, and convergence problems despite many positive aspects.

## 3. Research Methodology

This section is divided into three categories that will assist in understanding the review procedure and its ambition.

### 3.1. Planning of the Review

Three systematic advances are utilized that comprise the planning behind our work. First, based on efficacy and frequency of applicability on classifying HSIs, seven most recently used ML techniques have been chosen in this article for review, which establishes the operational relationship and compatibility with the issue of categorizing the land covers of a particular scene captured as HSI. Second, this relationship provides all the shortfalls and benefits of those methods and their potential possibilities. Finally, we identified the limitations of our present review work and how to rectify them in the future.

### 3.2. Conducting the Review

The entire review work has been conducted in the following steps:

(a) Collection of literature: The literature studies have been collected based on the keywords: “Hyperspectral image classification,” “Machine learning techniques,” “Deep learning techniques,” from the most relevant search engine, that is, Google (Google Scholar), which provides the scholarly articles for the concerned topic. These literature studies include Web of Science (WoS), Scopus, SCI, and SCIE-indexed and SCIE-related articles, both journals and conferences. Several methods are utilized throughout the literature that assist the classification of hyperspectral data, out of which ML techniques seem to be more convenient and promising.
(b) Screening: The collected research papers depict raw data, sorted categorically according to the chronological order of the ML techniques used over the periods. The screening was accomplished based on the following constraints:
  - Time Period: The studies published in the range of 2010–2021 are included in this work. Studies published before 2010 are not included.
  - Methodology: The studies on HSI's analytical operations (denoising, spectral unmixing, etc.) other than classifying the underlying land covers are rejected.
  - *Type*: The studies that deal with the hyperspectral images of a particular land scene are considered, discarding the medical hyperspectral imagery, water reservoir, etc.
  - Design of study: The studies comprising experimental outcomes and the elaboration of the models are accepted; other literary-based articles or review papers are only for primary knowledge gain.
  - The language used: The studies written in the English language are only considered.
Figure 1 represents the total number of the literary studies screened individually on each of the categories of chosen ML techniques in the form of pie-charts with a percent-wise pattern.  Figure 2 is a standard graphical depiction of the number of most recent articles that we screened for each chosen ML-based method in the period ranging from 2015 to 2021.
(c) Selection: Out of all the papers screened based on the abovementioned criteria, a few most eligible are handpicked. The selection has been made keeping specific parameters: the modeling strategy and algorithm and its suitability with the modern technological scenario. The final result is the corresponding overall accuracy (COA) for each dataset used, preferably journals with a good citation index.
(d) Analysis and inference: These selected papers are thoroughly reviewed to determine their contribution, restrictions, and future propositions. Based on this analysis, the deductions are drawn to show the pathway of further research.

### 3.3. Research Investigations (RI)

The analysis arises some of the queries:

  RI 1: What is the significance of traditional ML and DL for analyzing HSI?
  RI 2: How is ML/DL more impactful on HSI than other non-ML strategies?
  RI 3: What are the advantages and challenges faced by the researchers for the chosen ML/DL-based algorithm for HSI classification?
  RI 4: What are the emerging literary works of ML/DL on HSI classification in the year 2021?
  RI 5: How are ML- and DL-based hybrid techniques helping scientists in HSI classification?
  RI 6: What are the latest emerging techniques associated with addressing classifying HSIs?

### 3.4. Datasets

The HSI datasets are pre-refined and made publicly available for download and perform operations. There are six datasets that are described here in a concise manner:

- AVIRIS Indian Pines: This dataset was taken by airborne visible infrared imaging spectrometer (AVIRIS) sensor, on June 12, 1992. The scene captured here was Indian Pines test site in North-Western Indiana, USA, and contains an agricultural area exemplified by its crops of regular geometry and some irregular forest zones. It consists of 145 ∗ 145 pixels with a spectral resolution of 10 nm and a spatial resolution of 20 mpp and 224 spectral reflectance bands in the wavelength range 0.4–2.5 *μ*m, out of which 24 noisy bans are removed due to low signal-to-noise ratio. The scene contains 16 different classes of land covers.
- Salinas Valley: This scene was obtained by AVIRIS sensor over various agricultural fields of Salinas valley, California, USA, in 1998. The scene is characterized by a high spatial resolution of 3.7 mpp and a spectral resolution of 10 nm. The area is covered by 512 ∗ 217 spectral samples with a wavelength range of 0.4–2.5 *μ*m. Out of 224 reflector bands, 20 noisy bands are discarded due to water absorption coverage. The scene comprises 16 different land classes.
- Pavia Center: This scene was captured by a reflective optics system imaging spectrometer (ROSIS-03) sensor during a flight campaign over Pavia, northern Italy. It possesses 115 spectral bands, out of which only 102 are useful. Its spectral coverage is 0.43–0.86 *μ*m, with a spectral resolution of 4 nm and a spatial resolution of 1.3 mpp defined by 1096 ∗ 1096 pixels. There are 9 different land cover classes in the area.
- Pavia University: This scene was also captured by the same sensor at the same time as Pavia center, over the University of Pavia in 2001. It has the same structural features as the Pavia center, only contrasting in considering 103 bands out of 115 bands with a size of 610 ∗ 340 are taken after discarding 12 noisy bands. The scene contains 9 classes with urban environmental constructions.
- Kennedy Space Center: This scene was acquired by NASA AVIRIS sensor over Kennedy Space Center, Florida, USA, on March 23, 1996. It was taken from an altitude of approximately 20 kilometres, having a spatial resolution of 18 kilometres and a spectral resolution of 10 nm. The wavelength range of the scene is 0.4–2.5 *μ*m with the special size of 512 ∗ 614 pixels; 24 of 48 bands were removed for a low signal-to-noise ratio. The ground contains 13 predefined classes by the center personnel.
- Botswana*:* The scene was obtained by the Hyperion sensor placed on the NASA EO-1 satellite over Okavango delta, Botswana, South Africa, on May 31, 2001. It has a special resolution of 30 metres and a spectral resolution of 10 nm while taken at an altitude of 7.7 kilometres. Out of 242 bands containing 1476 ∗ 256 pixels, with a wavelength range of 400–2500 nm, 97 bands are considered to be water-corrupted and noisy; hence, 145 remaining are useful. The scene comprises 14 land cover classes.

## 4. Machine Learning-Based Techniques for HSI Classification

ML technologies are not only intelligent and cognitive, but also their accuracy is skyrocketing due to their embedded mechanical abilities such as extraction, selection, and reduction of joint spatial-spectral features as well as contextual ones [24–26]. Moreover, the hidden dense layers with various allocated functions of the extensive networks work as intelligent learners by creating dictionaries or learning spaces to store deterministic information and then separate the landcover classes through its classification units [27–29]. The latest ML techniques that assist in classifying the hyperspectral data, that is, SVM, SRC, ELM, MRF, AL, DL, and TL, are shown categorically in Figure 3 and are discussed hereafter in detail.

### 4.1. Support Vector Machine (SVM)

SVM is an innovative pattern-recognition technique rooted in the principle of statistical learning. The rudimentary concept of SVM-based training can unravel the ideal linear hyperplane so that the predicted classification error is mitigated, be it for binary or multiclass purposes [30], as depicted in Figure 4. For linearly separable binary classification, let (*x*_*i*_, *y*_*i*_) be the standard set of linearly separating samples with *x* ∈ (*R*)^*N*^ and *y* ∈ {−1, +1}. The universal formula of linear decision function in n-dimensional space with the classification hyperplane is

(1) $$\begin{array}{c} g\left(x\right)=w^{T}.x+b=0, \end{array}$$

where *w* is the weight directional vector and *b* is the slope of the hyperplane. A separating hyperplane with margin 2/||*w*|| in the canonical form must gratify the following constraints:

(2) $$\begin{array}{c} y_{i}\left[\left(w^{T}.x_{i}\right)+b\right]\geq 1. \end{array}$$

For multiclass scenarios, we presumably transform the datapoints to *S*, a probable infinite-dimensional space, by a mapping function *ψ* defined as *ψ*(*x*) = (*x*_1_^2^, *x*_2_^2^, √2*x*_1_*x*_2_), **x** = (*x*_1_, *x*_2_). Linear operations performed in S resemble nonlinear processes in the original input space. Let *K*(*x*_*i*_, *x*_*j*_) = *ψ*(*x*_*i*_)^T^*ψ*(*x*_*j*_) be the kernel function, which remaps the inner products of the training dataset.

Constructing SVM requires values of the constants, that is, Lagrange's multipliers, *α* = (*α*_1_,…, *α*_*N*_) so that

(3) $$\begin{array}{c} P\left(\alpha \right)=\sum_{i=1}^{N}\alpha_{i}-\frac{1}{2}\;\sum_{i,j=1}^{N}\alpha_{i}\alpha_{j}y_{i}y_{j}\;K\left(x_{i}\;.x_{j}\right). \end{array}$$

is maximized with the constraints with respect to *α:*

(4) $$\begin{array}{c} \sum_{i=1}^{N}\alpha_{i}y_{i}=0,\;\alpha_{i}\geq 0\text{ for all }\alpha_{i}. \end{array}$$

Because most *α*_*i*_ are supposedly equal to zero, samples conforming to nonzero *α*_*i*_ are support vectors. Conferring to the support vectors, the modified optimally ideal classification function is

(5) $$\begin{array}{c} f\left(x\right)=\sum_{i=1}^{N}\alpha_{i}y_{i}K\left(x_{i}.x_{j}\right)+b. \end{array}$$

The application of SVM for classifying HSI started two decades ago [31, 32]. Focusing on the potentially critical issue of applying binary SVMs [33], fuzzy-based SVM [34] as fuzzy input-fuzzy output support vector machine (F2-SVM), SVM evolved to dimensionality reduction and mixing of morphological details [35]. It also assisted particle swarm optimization (PSO) [36] and wavelet analysis with semi-parametric estimation [37], as the classifier “wavelet SVM” (WSVM).  Table 1 summarizes the research carried out so far for the classification purpose of HSI using SVM.

### 4.2. Sparse Representation and Classification (SRC)

Sparse method depends on dictionary learning that enhances and rectifies the values of parameters based upon the current training observations while accumulating the knowledge of the previous observations prior. It then generates the sparse coefficient vector using sparse coding. This method is supremely efficient as it embeds dictionary learning to extract rich features embedded inside the HSI dataset. SR can classify images pixelwise by representing the patches around the pixel with a linear combination of several elements taken from the dictionary. The generalization of SRC called multiple SRC (mSRC) has three chief parameters—patch size, sparsity level, and dictionary size. Dictionary learning is the first step for sparse, using K-SVD algorithm. Let *Y* = [*y*_1_, *y*_2_,…, *y*_*N*_] be a matrix of L2-normalized training samples *y*_*i*_ ∈ *R*^*m*^ [45–47].

The size of patches around the pixel is

(6) $$\begin{array}{c} \underset{D,B}{\min}{\left\|Y-\text{DB}\right\|}_{F}^{2}\text{ such that }\left\|b_{i}\right\|\;0\leq S,\text{for all }i, \end{array}$$

where *D* is a member of **R**^*mXn*^ is the learned over a complete dictionary, with *n* > *m* atoms, *B* = [*b*_1_, *b*_2_,…, *b*_*m*_] represents the matrix of corresponding sparse coding vectors *b*_*i*_ ∈ **R**^*n*^, and ∣∣·∣∣_*F*_ is the Frobenius norm. Sparsity *S* limits the number of nonzero coefficients in each *b*_*i*_. The next step sparse coding is provided with dictionary *D* and represents *y* as a linear combination of *y* = *D*$\overset{\wedge }{b}$ where $\overset{\wedge }{b}$ is sparse. For the final classification step, suppose for each class *j* ∈ {1,…, *M*} of an image, a dictionary *D*_*i*_ is trained. Then, the classification of a new patch *y*_test_ is achieved by estimating a representation error. The class assignments rule [47] is calculated through a pseudoprobability measure *P*(*C*_*j*_) for each class error *E*_*j*_ as

(7) $$\begin{array}{c} j*\;=\;\underset{j}{\arg\max}P\left(C_{j}\right),\;\text{where, }P\left(C_{j}\right)=\frac{1}{M-1}\frac{\sum_{k=1,k\neq j}^{M}E_{k}}{\sum_{k=1}^{M}E_{k}}. \end{array}$$

mSRC obtains residuals of disjoint sparse representation of *y*_test_ for all classes *j*. Each dictionary *D*_j_ is updated by eliminating nonzero atoms from ${\overset{\wedge }{b}}_{j}$ after each of *k* iterations and *y*_test_ is assigned to the class, using *Q* total iterations:

(8) $$\begin{array}{c} D_{j}\;=\underset{j}{\text{argmax}}\sum_{k=1}^{Q}P_{k}\left(C_{j}\right). \end{array}$$

Sparse representation is an essential and efficient machine-dependent method in many areas, including denoising, restoration, target identification, recognition, and monitoring. It may grow even more vital when associated with logistic regression, adaptivity, and super-pixels to extricate the joint features globally and locally. SR has a very high potential of being associated with methods such as PCA, ICA, Markov random fields, conditional random fields, extreme learning machines, and DL methods such as CNN and graphical convolutional network.  Table 2 gives a summary of the research performed so far for the classification purpose of HSI employing SRC.

### 4.3. Markov Random Field (MRF)

MRF describes a set of random variables satisfying Markov probability, depicted by undirected graphs. It is similar to the Bayesian network but, unlike it, undirected and cyclic. An MRF is represented as a graphical model of a joint probability distribution defined in Figure 5. The undirected graph of MRF, *G* = (*V*, *E*), in which *V* is the nodes representing random variables.

Based on the Markov properties [57], the neighborhood set *N*_*c*_ of a node *c* is defined as

(9) $$\begin{array}{c} N_{c}=\left\{c\in V|\left(c,d\right)\in \;E\right\}. \end{array}$$

The conditional probability of *Y*_*c*_ decides the joint distribution of *Y* as

(10) $$\begin{array}{c} P\left(Y_{c}|Y_{v}-Y_{c}\right)=P\left(Y_{c}|Y_{\text{Nc}}\right). \end{array}$$

To prosper the construction, the graph **G** absorbs a Gibbs distribution all over the maximum cliques (*C*) in **G**:

(11) $$\begin{array}{c} P\left(y\right)=\prod_{mЄC}\psi_{m}\left(y_{m}\right)\;\;=\frac{1}{Z}\;e^{-1/T\sum_{mЄC}V_{m}\left(y_{m}\right)}, \end{array}$$

where *Z* is the partition function. Therefore, equation (11) can be rewritten as

(12) $$\begin{array}{c} P\left(y\right)=\;\frac{1}{Z}e^{-1/TU\left(y\right)}, \end{array}$$

where *T* is the temperature, whose value is generally 1, and *U*(*y*)=∑_*mЄC*_*V*_*m*_(*y*_*m*_) represents the energy.

Markov models depict the stochastic method that is represented by a graph made of circles has an acute advantage of not considering the past states for all upcoming future states for a random alterable dataset such as HSIs. The variants of Markov random fields are adaptive, hierarchical, cascaded, and probabilistic, a blend of Gaussian mixture model, joint sparse representation, transfer learning, etc., whose outcomes are pretty victorious. Hidden Markov random fields are highly suitable for the unsupervised classification of HSIs where the model parameters are estimated to make each pixel belong to its appropriate cluster [58], leading to the precise classification.  Table 3 lists out the research carried out so far for the classification purpose of HSI employing MRF.

### 4.4. Extreme Learning Machine (ELM)

An efficacious learning algorithm based on single hidden layer feedforward neural network (SLFNN), it is applied to classify patterns and regression. Let (*x*_i_, *p*_i_) ∈ **R**^*n*^*X ***R**^*m*^ be N arbitrarily perceptible samples where *x*_*i*_ = [*x*_*i*1_,…, *x*_*in*_]^T^ ∈ **R**^*n*^ and *p*_*i*_ = [*p*_*i*1_,…, *p*_*im*_]^T^ ∈ **R**^*m*^ [72]. The standard SLFNN having $\overset{\wedge }{N}$ hidden nodes and *f*(*x*) as activation function is approached mathematically as

(13) $$\begin{array}{c} \sum_{i=1}^{\hat{N}}\alpha_{i}f_{i}\left(x_{i}\right)=\sum_{i=1}^{\hat{N}}\alpha_{i}f\left(w_{i}.x_{j}+b_{i}\right)=O_{j};\;j=1,\ldots ,N. \end{array}$$

Here, *w*_*i*_ = [*w*_*i*1_,…, *w*_*in*_]^T^ gives the weight vector establishing the connection between input nodes and *i*^th^ is the hidden node and *α*_*i*_ = [*α*_*i*1_,…, *α*_*im*_]^T^ represents the weight vector connecting between output node *O*_*j*_ with the *i*^th^ hidden node, and *w*_*i*_.*x*_*j*_ represents the inner product. The zero error for *N* samples can be written in the matrix form as *Aα* = *P*, where *A* (*w*_1_,…, $w_{\hat{N}}$, *b*_1_,…, $b_{\hat{N}}$, *x*_1_,…, *x*_*N*_) is the neural network hidden layer output matrix, and the *i*^th^ is hidden node output with respect to *x*_1_,…, *x*_*N*_; the *i*^th^ column of *A* represents *x*_*N*_ inputs. The training of SLFNN is based on finding specific *α*, *w*_*i*_, and *b*_*i*,_ (*i* = 1,…, $\hat{\text{N}}$) [73] such that

(14) $$\begin{array}{c} \left\|A\left(w_{1},\ldots ,w_{\hat{N}},\;b_{1},\ldots ,\;b_{\hat{N}},\;x_{1},\ldots ,\;x_{N}\right)\alpha -P\right\|=\underset{w,\alpha ,\;b}{\min}\left\|A\left(w_{1},\;\ldots ,w_{\hat{N}},b_{1},\;\ldots ,\;b_{\hat{N}},\;x_{1},\;\ldots ,\;x_{N}\right)\alpha -\;P\right\|. \end{array}$$

This equation denotes the cost function with a depreciation. By using gradient-based algorithms, the set of weights (*α*_*i*_, *w*_*i*_) and biases *b*_*i*_ are attuned with epochs as

(15) $$\begin{array}{c} w_{k}=w_{k-1}-\eta \frac{\delta U\left(W\right)}{\delta W};\\ U=\sum_{k=1}^{N}{\left(\overset{\hat{N}}{\underset{j=1}{\sum }}\alpha_{j}f\left(w_{j}.\;x_{k}+b_{j}\right)-P_{k}\right)}^{2}. \end{array}$$

The learning rate *η* must be accurate for better convergence and $\overset{\wedge }{N}$ << N for better generalization performance.

Extreme learning methods proposed overcoming the disadvantage of a single hidden layer feedforward neural network and improving learning ability and generalization performance. It is a supervised method but is highly recommended to get an extension to its semi-supervised and unsupervised versions for dealing with the huge amount of data such as HSIs, which are primarily unlabeled and suffering from lack of training samples. Great potential lies with its other variants than those mentioned here, [74] of ELM, like two-hidden layer ELM, multilayer ELM, feature mapping-based ELM, incremental ELM, and deep ELM to become superior and achieve victorious precision in classifying HSIs.  Table 4 underneath provides the summary of the research executed so far for the classification purpose of HSI utilizing ELM.

### 4.5. Active Learning (AL)

It is a special type of the supervised ML approach to build a high-performance classifier while minimizing the size of the training dataset by actively selecting valuable data points. The general structure of AL can be understood from Figure 6. There are three categories of AL—stream-based selective sampling, that is, where each unlabeled dataset is enquired for a certain label whether to assign a query or not; pool-based sampling; that is, the whole dataset is under consideration before selecting the best set of queries; and membership query synthesis; that is, it involves data augmentation to create user selected labeling. The decision to select the most informative data points depends on the uncertainty measure used in the selection. In an active learning scenario, the most informative data points are those the classifier is least sure about. The uncertainty measures for datapoints *x* [88] are

*Least Confidence (LC)*: responsible for selecting the classifier's data point is least certain about the chosen class. With *y*^∗^ as the most likely label sequence and ф as the learning model, LC is represented as
  (16) $$\begin{array}{c} S_{\text{LC}}\left(x\right)=1-P\left(y*|x,\;ф\right). \end{array}$$
*Smallest Margin Uncertainty (SMU)*: Represents the difference between classification probability of the most likely class (*y*_1_∗) and that of the second-best class (*y*_2_∗), written mathematically as:
  (17) $$\begin{array}{c} S_{\text{SMU}}\left(x\right)=P_{ф}\left(y_{1}*|x\right)-P_{ф}\left(y_{2}*|x\right). \end{array}$$
*Largest Margin Uncertainty (LMU)*: Represents the difference between classification probability of most likely class (*y*_1_∗) and that of the least likely class (*y*_min_), written mathematically as:
  (18) $$\begin{array}{c} S_{\text{LMU}}\left(x\right)=P_{ф}\left(y_{1}*|x\right)-P_{ф}\left(y_{\min}*|x\right). \end{array}$$
*Sequence Entropy (SE)*: Detects the measure of disorder in a system; higher the entropy implies a more disordered condition. The denotation of SE is
  (19) $$\begin{array}{c} S_{\text{SE}}\left(x\right)=-\sum_{\overset{\wedge }{y}}P\left(\overset{\wedge }{y}|x;ф\right)\log\;P\left(\overset{\wedge }{y}|x;ф\right), \end{array}$$
with $\hat{y}$ ranging over all possible label sequences for input *x*.

Although not considered customary and coherent, AL is pretty much capable of reducing human effort, time, and processing cost for a large batch of unlabeled data. This method relies on prioritizing data that needs to be labeled in a huge pool of unlabeled data to have the highest impact on training. A desired supervised model keeps on being trained through active queries and improvising itself to predict the class for each remaining data point. AL is advantageous for its dynamic and incremental approach to training the model so that it learns the most suitable label for each data cluster [89].  Table 5 lists out the research performed so far for the classification purpose of HSI using AL.

### 4.6. Deep Learning (DL)

Deep learning is the most renowned ML technology in application and accuracy terms. Although it is considered the next tread of ML, it also lends concepts from artificial intelligence. DL is the mother of algorithms that resemble human brain simulations, that is, creativity, enhanced analysis, and proper decision-making, based on pure or hybrid large networks for any given real-life problem. It has enhanced the throughput of computer-based, especially unsupervised snags for the practical technology-based applications such as automated translation of machines, image reconstructions and classifications, computer vision, and automated analysis. [104] The basic structure of any DL model possesses a three-type-layered architecture: it contains one input layer through which input data are fed to the next layer(s) known as the intermediate hidden layer responsible for all the computations based on the problem given, which passes its generated data to the final layer, that is, the output layer, which provides the desired ultimate output. The steps involved in DL models are as follows: having proper knowledge and understanding of the problem, collecting the input database, selecting the most appropriate algorithm, training the model with the sample source database, and finally testing the target database [105].

DL models are more efficient and advantageous over other ML models due to the following reasons [19]:

1. The capability to extract hidden and complicated structures from raw data is inextricably linked to their ability to represent the internal representation and generalize any form of knowledge.
2. They have a wide range of data types that they can accommodate, for example, 2D imagery data and complex 3D data such as medical imagery and remote sensing. In addition, they can use HSI data's spectral and spatial domains in both standalone and linked ways [106–108].
3. They provide architects a lot of versatility in terms of layer types, blocks, units, and depth.
4. Furthermore, its learning approach can be tailored to various learning strategies, from unsupervised to supervised, with intermediate strategy.
5. Additionally, developments in processing techniques, including batch partitioning and high-performance computation, especially on distributed and parallel architecture, have enabled DL models to find better opportunities and solutions when coping with enormous volumes of data [109].

The models that are broadly used for HSI classification are described as follows.

(a) Autoencoder (AE): AEs are the fundamental unsupervised deep model based on the backpropagation rule. AEs consist of two fragments: encoder, connecting the input vector to the hidden layer by a weight matrix; decoder, formed by the hidden layer output via a reconstruction vector tied by a specific weight matrix. SAEs are AEs with multiple hidden layers where the production of every hidden layer is fed to the successive hidden layer as input. It comprises three steps: (1) first AE trained to fetch the learned feature vector; (2) the former layer's feature vector is taken as input to the next layer, and this process is redone till the completion of training; (3) backpropagation is used after all the hidden layers have been trained to reduce the cost function and to update the weights is done with a named training set to obtain fine-tuning [110]. The architecture of SAE is depicted in Figure 7.
Let *x*_*n*_ ∈ **R**^*m*^; *n* = 1, 2,…, *N* represent the unlabeled input dataset, *E*_*n*_ be the hidden encoder vector computed by *x*_*n*_, and *y*_*n*_ be the decoder vector of the output layer [111].
  (20) $$\begin{array}{c} \text{Encoder: }E_{n}=g\left(W_{i}x_{n}+b_{i}\right); \end{array}$$
*g*-> encoding function, *W*_*i*_-> encoder weight matrix, *b*_*i*_-> encoder bias vector.
  (21) $$\begin{array}{c} \text{Decoder: }y_{n}=f\left(W_{j}E_{n}+b_{j}\right); \end{array}$$
*f*-> decoding function, *W*_*j*_-> decoder weight matrix, *b*_*j*_-> decoder bias vector.
The reconstruction error in SAE is denoted as
  (22) $$\begin{array}{c} \Phi \left(\Theta \right)=\;\arg\underset{\theta ,\theta^{\prime }}{\min}\frac{1}{N}\sum_{k=1}^{N}L\left(x^{k},y^{k}\right),\text{where the Loss function is }L\left(x^{k},y^{k}\right)={\left\|x-y\right\|}^{2}. \end{array}$$
AEs are unsupervised neural networks that embed several convolutional hidden layers based on nonlinear activation functions and transformations [112]. There are high risks of data loss during training, but it handles the model well for specific data types through specialized training. There are AEs for every purpose such as convolutional, sparse, variational, deep, contractive, and denoising applied for data compression, noise removal, feature extraction, image augmenting, and image coloring. AE inevitably provides a vast platform for further research on its various applicability and its capability to participate in hybridization.  Table 6 describes a few research works in the aspect of AEs.
(b) *Convolutional Neural Network (CNN)*: It is a famous deep neural network that works like a human visual cortex with many interconnected layers applied widely in image, speech, and signal processing. It assigns learnable and modifiable weights and biases to the input image to identify various objects or patterns with differentiable features. As shown in Figure 8, each layer of CNN possesses filtering capabilities with ascending complexities: the first layer learns filtering corners and edges; intermediate layers learn object parts filtering; and the last layer learns filtering out the entire object in different locations and shapes. The comparison between the layers in terms of several parameters is shown in Table 7. It consists of four layers [117, 118]:
  (1) *Convolution*: This operation is the cause of the naming of CNN, that is, a dot product of the original pixel values with weights identified in the filter or kernel of the image. The findings are compiled into one number representing all the pixels found in the filter. Assuming **I** be the hyper-input-cube of dimension *p* × *q* × *r* where *p* × *q* denotes the spatial size of **I** with *r* number of bands, and *i*_*k*_ is the *k*th feature map of **I**. Let *d* number of filters be present in each convolutional layer, and weight *W_m_* and bias *b_m_* represent the *m*th filter. The *m*^th^ convolutional layer output with transformation function *g* is denoted as
    (23) $$\begin{array}{c} Y_{m}\;=\sum_{k=1}^{r}g\left(i_{k}.W_{m}+b_{m}\right);m=1,2,\ldots ,d. \end{array}$$
  (2) *Activation*: The convolution layer produces a matrix significantly smaller than the actual image. The matrix is passed through an activation layer (generally rectified linear unit, aka ReLU), adding nonlinearity that enables the network to train itself through backpropagation.
  (3) *Pooling*: It is the method of even more downsampling and reduction of the matrix size. A filter is applied over the results obtained by the previous layer and chooses a number from each set of values (generally the maximum, the max-pooling), which allows the network to train much more quickly, concentrating on the most valuable information in each image feature. For an *m* × *m* square window neighbor *S* with *N* elements and *z*_*ij*_ activation value concerning (*i*, *j*) location, the average pooling is formulated as
    (24) $$\begin{array}{c} T\;=\frac{1}{N}\sum_{\left(i,j\right)\epsilon S}z_{\text{ij}}. \end{array}$$
  (4) *Fully Connected (FC)*: A typical perceptron structure with multilayers. The input is a single-dimensional vector representing the output of the layers above. Its output is a probability list for the various possible labels attached to the image. Classification decision is the mark that receives the highest likelihood. It is mathematically represented with transformation function *g*, for *N* samples of inputs with *X*″ and *Y*″ being the outputs having *W* being the weight matrix and *b*, the bias constant, is as follows:
    (25) $$\begin{array}{c} Y^{\prime \prime }=\sum_{j=1}^{N}g\left(\text{WX}{}^{\prime \prime }+b\right). \end{array}$$
  CNN is the most method-in-demand and widely explored model among all DL models. The functional unit of convolutional layers is kernels that expertise in extricating the most relevant and enriched spatial and spectral features from the given dataset through automated filtering by convolution operation [119]. It provides an intense description of the whereabouts of CNNs. The most popular ones are attention-based CNN, ResNet, CapsNet, LeNet, AlexNet, VGG, etc. Some of them are still unexplored yet in classifying HSI. The detailed research work on CNN for dealing with HSI classification is listed in Table 8.
(c) *Recurrent Neural Network (RNN):* DL is a very efficient approach that follows a sequential framework with a definite timestamp *t*. “Recurrent” refers to performing the same task for each sequence element, with the output depending on the preceding computations. In other words, they have a “memory” that enfolds information about the calculation so far type of neural network, and the output of a particular recurrent neuron is fed backward as input to the same node, which leads the network to efficiently predict the output, represented in Figure 9, where RNN unrolls, that is, show the complete sequence of the entire network structure neuron by neuron. It consists of the following steps:
  (1) **X** = […, *x*_*t*−1_, *x*_*t*_, *x*_*t*+1_,…] be the input vector, where *x*_*t*_ represents input at timestamp *t*.
  (2) *h*_*t*_ is the “memory of the network,” the hidden state at timestamp *t*. Preliminarily, *h*_−1_ is initialized to zero vector to calculate the first hidden step. *h*_*t*_ being the current step is calculated based on previously hidden step *h*_*t*−1_, formulated by [132]
    (26) $$\begin{array}{c} h_{t}=f\left({\text{Px}}_{t}+{\text{Wh}}_{t-1}\right), \end{array}$$
  where *f* denotes a function of nonlinearity, that is, tanh or ReLU, and *W* be the weight vector.
  (3) **Y** = […, *y*_*t*−1_, *y*_*t*_, *y*_*t*+1_,…] be the output vector, where *y*_*t*_ represents input at timestamp *t*, generally a softmax function: *y*_*t*_ = softmax(*Q h*_*t*_).
  RNN is an efficient deep model with large potential. The recurrence looping structure acquainted with RNN enables it to store relevant information about spatial-spectral relationships between the pixels and neighbors. There are several RNN architectures based on inputs/outputs as stated in [133], and based on LSTM, there are five categories [134]. These variates can be well utilized in collaboration with other DL methods such as MRF and PCA to find their accuracy.
  The literature studies based on RNN are cataloged in Table 9.
(d) Deep Belief Network (DBN): DBNs are formed by greedy stacking and training restricted Boltzmann machines (RBMs), an unsupervised learning algorithm based on “contrastive divergence.” For neural networks, RBMs suggest taking a probabilistic approach and are thus called stochastic neural networks. Each RBM is made of three parts: a visible unit (input layer), an invisible unit (hidden layer), and a bias unit. The general structure of a DBN is depicted in Figure 10.
For a DBN, the joint distribution of input vector, *X* with *n* hidden layers *h*_*n*,_ is defined as [137]
  (27) $$\begin{array}{c} P\left(X,h_{1},\ldots ,h_{n}\right)\;=\left(\overset{n-2}{\underset{i=0}{\prod }}P\left(h_{i}|h_{i+1}\right)\right).P\left(h_{n-1},\;h_{n}\right), \end{array}$$
where *X* = *h*_0_, *P*(*h*_*i*−1_, *h*_*i*_) is the conditional distribution of the visible units on the hidden RBM units at level *i* and *P*(*h*_*n*−1_, *h*_*n*_) is the hidden-visible joint distribution in top-level RBM. DBN has two phases: the pretraining phase depicts numerous layers of RBM, and fine-tuning phase is simply a feedforward NN.
DBN is the graphical representation that is generative; that is, it creates all distinct outcomes that can be produced for the particular case and learn to disengage a deep hierarchical depiction of the sample training data. DBNs are structurally more capable than RNNs as they lack loops, are pretrained in an unsupervised way, and are computationally eminent for particularly classification problems. Minor modifications or collaborations can improvise DBNs functionally and accuracy.  Table 10 depicts a list of works done on DBN.
(e) Generative Adversarial Network (GAN): One of the most recent DL models that are rapidly growing its footsteps in the area of technical research. The GAN model is trained using two kinds of neural networks: the “generative network” or “generator” model that learns to generate new viable samples and the “discriminatory network” or “discriminator,” which learns to discriminate generated instances from existing instances. Discriminative algorithms seek to classify the input data, which is given as a collection of certain features; the algorithm maps feature on labels [140]. In contrast, generative algorithms attempt to construct the input data, which is given with a set of features, and it will not classify it, but it will attempt to create a feature that matches a certain label. The generator tries to get better at deluding the discriminator during the training, and the discriminator tries to grab the counterfeits generated by the generator. Thus, the training procedure is termed adversarial training. The generator and discriminator should be trained against a static opponent, keeping the discriminator constant while training the generator and keeping the generator constant when training the discriminator. That helps to understand the gradients better.

In a GAN model, say *D* and *G* denote the discriminator and the generator units that map a noise data space *θ* to real and original data space *x*, respectively. *G*(*θ*) denotes the fake output generated by *G*, and *D*(*y*), and *D*(*G*(*θ*)) are *D*'s output for real and fake training samples, respectively. *P*_*θ*_(*θ*) and *P*_*d*_(*y*) represent the input model distribution and original data distribution, respectively, when *θ*∼*P*_*θ*_ [141] as shown in Figure 11.

(28) $$\begin{array}{c} \text{The loss function for }D:L^{\left(D\right)}=\max\left[\log\left(D\left(y\right)\right)+\log\;\left(1-D\left(G\left(\theta \right)\right)\right)\right]. \end{array}$$

(29) $$\begin{array}{c} \text{The Loss function for }G:L^{\left(G\right)}=\min\left[\log\left(D\left(y\right)\right)+\log\;\left(1-D\left(G\left(\theta \right)\right)\right)\right]. \end{array}$$

Combining equations (28) and (29), the total loss of the entire dataset represented by the min-max value function is given by

(30) $$\begin{array}{c} \underset{G}{\min}\underset{D}{\max}\;V\left(D,G\right)=\;\underset{G}{\min}\underset{D}{\max}\left(E_{y}∼P_{d}\left(y\right)\left[\log\left(D\left(y\right)\right)\right]+E_{\theta }∼P_{\theta }\left(\theta \right)\left[\log\left.\left(1-D\left(G\left(\theta \right)\right)\right)\right]\right.\right). \end{array}$$

GAN is a generative modeling neural network architecture based on the concept of adversarial training that utilizes a model to build new instances that are conceivably derived from an existing sample distribution. Hence, GANs are new favorites for classifying HSIs as they compensate for the lack of data problem and classify the data in a pro manner. There are several types of GANs—conditional GAN, vanilla GAN, deep convolutional GAN (simple type); and Pix2Pix GAN, CycleGAN, StackGAN, and InfoGAN (complex type) [142]. These may be very useful for images like HSIs as they can deal with related issues. The research works based on the GAN are listed in Table 11.

### 4.7. Transfer Learning (TL)

It is the most current hot topic in interactive learning, and there are more to it to be explored. It is an approach where information gained is transferred in one or more source tasks and is used to enhance the learning of a similar target task. TL can be represented diagrammatically by Figure 12 and mathematically shown as follows:

Domain, **D**, is represented as {**X**, *P*(*X*)}, *X* = {*x*_1_,…, *x*_*n*_}, *x*_*i*_ ∈ **X**; **X** denotes the feature space, and *P*(*X*) symbolizes the marginal probability of sample data point *X* [149].

Task **T** is depicted as {**Y**, *P*(*Y*|*X*)} = {**Y**, Φ}, *Y* = {*y*_1_,…, *y*_*n*_}, *y*_*i*_ ∈ **Y**; **Y** is the label space, Φ is the prognostic objective function, having learned form (feature vector, label) couples, (*x*_*i*_, *y*_*i*_); *x*_*i*_ ∈ **X**, *y*_*i*_ ∈ **Y**, and calculated as the conditional probability.

Also, for every feature vector in **D**, Φ predicts its corresponding label as Φ(*x*_*i*_) = *y*_*i*_.

If **D**_*S*_ and **D**_*T*_ be the source and target domains, **T**_*S*_ and **T**_*T*_ be the source and target tasks, respectively, with **D**_*S*_ ≠ **D**_*T*_ and **T**_*S*_ ≠ **T**_*T*_. TL objectifies to learn *P*(*Y*_*T*_|*X*_*T*_), that is, the target conditional probability distribution in **D**_*T*_ with knowledge obtained from **D**_*S*_ and **T**_*S*_.

Traditional learning is segregated and solely based on particular tasks, datasets, and different independent models working on them. No information that can be converted from one model to another is preserved, but on the contrary, TL possesses the human-like capability of transferring knowledge; that is, knowledge can be leveraged from priorly trained models to train new models, the process of which is faster, more accurate, and with the limited amount of training data.  Table 12 represents a brief detail about the research works on transfer learning.

## 5. Discussion

Based on the reviewed articles, we can draw the desired inferences that provide answers to the investigative questions mentioned in Section 2 and show the clear motive and benefits of this review.

*RI 1: What is the significance of traditional ML and DL for analyzing HSI?*

Ans: Hyperspectral data have certain restrictions, as cited in Section 1. Statistical classifiers initially addressed them, but the operations and analysis became much easier and more accurate after the invention of ML/DL strategies in a machine-dependent way [155, 156]. The general advantages that researchers were provided by the ML/DL algorithms while dealing with HSIs are as follows: (i) easy dealing with high-dimensional data, that is, troubles of Hughes phenomenon removed [115, 125]; (ii) equally manipulative to labeled and unlabeled samples [99, 150]; (iii) precise and the meticulous choice of features [51, 127]; (iv) high-end-precise models to deal with real hypercubes, hence top-notch classification accuracy [119, 154]; v) removes overfitting, noises, and other hurdles to a much greater extent [120, 147]; (vi) embedded spatial-spectral feature extraction and selection units [119, 133]; (vii) mimics human brain to solve multiclass problems [136, 138].

*RI 2: How are ML/DL more impactful on HSI than other non-ML strategies?*

Ans: The initial discovery of hyperspectral data has suffered due to its limitations. In the preliminary research stage, the scientists followed the traditional methodology for classifying HSIs, that is, preprocessing (if required), extraction, and selection of discriminative characteristics and then ran a classifier on those features to identify the land cover groups. Hence, they emphasized the feature extractor techniques such as PCA [9], ICA [10], and wavelets [13], assisted by some basic random classifiers such as extended morphological profiles [2, 157], NN [158, 159], logistic regression [160], edge-preserving filters [10, 161], density functions/matrices [162], and Bayes law of classification [163, 164]. These classic mathematics-oriented techniques were not enough to deal with such a huge amount of data like HSI, as they were simple in structure and design and easy to implement. It also could not predict well enough the multiclass problems, which is very much required for a dataset like HSI, whose land covers belong to multiple classes of regions. Also, these methods were not accurate in feature selection and extraction or dealing with the storage of such bulk data. These reasons made researchers struggle to analyze properly, process, and classify HSIs. On the contrary, the advancements of ML/DL technologies have opened a broad gateway of research that researchers are still exploring and combining with different groupings to address the HSI classification problem in real life, dealing with the limitations mentioned above [26, 131]. The tabular depiction of the advantages and disadvantages of the ML and non-ML strategies applied for HSI classification is shown in Table 13.

*RI 3: What are the advantages and challenges faced by the researchers for the chosen ML/DL-based algorithm for HSI classification?*

Ans: We added the advantages and challenges of the ML- and DL-based techniques in Table 13.

*RI 4: What are the emerging literary works of ML/DL on HSI classification in the year 2021?*

Ans: In the ongoing years, 2021 seems to be more promising in terms of technical advancements for the problem concerned. New techniques are emerging, along with hybrid ones, to solve the issue to a whole new level, the methodologies' accuracy to be described. Recent work on MRF with a band-weighted discrete spectral mixture model (MRF-BDSMM) in a Bayesian framework has been proposed in [165], an unsupervised adaptive approach to accommodate heterogeneous noise and find the abundant labeled subpixels to extricate joint features. A collaboration of Kernel-based ELM with PCA, local binary pattern (LBP), and gray-wolf optimization algorithm (PLG) is proposed as novel methodologies. They help reduce huge dimensions, seek global and local-spatial features, and optimize the KELM parameters to obtain the class labels [166]. A variant of SRC is proposed in [167], dual sparse representation graph-based collaborative propagation (DSRG-CP) that separates spatial and spectral dimensions with the respective graph to improve the labeling scheme limited samples by collaborating the outcomes. AL has been one of the hot topics so far, as it integrates with a Fredholm kernel regularized model (AMKFL) that enables better labeling than manual ones, even for noisy images [168]. It ties with DL with the augmentation of training samples to label the uncertain hypercubes (ADL-UL) accurately [169], facilitates iterative training sample augmentation by expanding the hypercubes and adds discriminative joint features (ITSA-AL-SS) [170], extracts local unique spatial multiscale characteristics from the super-pixels (MSAL) [171]. A novel idea of attention-based CNNs is proposed in [172, 173], the former (SSAtt-CNN) collides two attention subnetworks—spatial and spectral with CNN as the base, and the latter (FADCNN) is a dense spectral-spatial CNN with feedback attention technique that perfectly poses the band weights for better mining and utilization of dominant features. GAN is one the most exploited methods to date, and [174] proposes the full utilization of shallow features from the unlabeled bands through a multitasking network (MTGAN); in [175], the discriminator is based upon capsule network and convolutional long short-term memory to extricate less visible features and integrates them to build high-profile contextual characteristics (CCAPS-GAN); 1D and 2D CapsGAN together form a dual-channel spectral-spatial fusion capsule GAN (DcCaps-GAN) shown in [176]; and generative adversarial minority oversampling for 3D-hypercubes (3D-HyperGAMO) is depicted in [177] that focuses on the minor class features using existing ones to label and classify them properly.

*RI 5: How are ML- and DL-based hybrid techniques helping scientists in HSI classification?*

Ans: Since the dawn of the emergence of HSIs, it has suffered many hurdles in its path of analysis and information extraction. The maximum number of highly correlated bands and the high spatial-spectral features signature by the electromagnetic spectrum embedded in it are always considered a traction matter. Thus, finding an appropriate technology for the classification of such interconnected and hugely confined featured high-dimensional images is a very tedious and strenuous matter. The classification methods chosen so far have been mostly limited to supervised. The requirement of a sufficient number of quality-labeled data and unsupervised, in which the lack of coherence between the spectral clusters and the target regions, causes the failure in obtaining the desired accuracy. A semi-supervised method is needed to overcome such problems as a combination of supervised and unsupervised methods, named the hybrid method. A hybrid method is always advantageous in robustness and flexibility towards the high-dimensional data.

The hybrid methods have the following benefits:

- Specifically designed to overcome the limitations and take advantage of the methodologies involved in the concerned hybrid to achieve a deep, rich, and insightful conclusion (general).
- Addressing and resolving multiple issues regarding the handling and analyzing the HSI data, at a time, depending upon the methods that are chosen for mixing/hybridizing [179–183].
- Coherence in time, space, and cost complexities [184–186].
- Better interpretability, quality, effectivity leading to the construction of a more refined framework [180, 182, 183, 187–194].
- Deterministic spectral, spatial, and contextual feature extraction, reduction, and selection, and combining them to achieve desired accuracy and performance [182, 183, 187, 188, 195–197].

ML, being a standard versatile technology, can merge with traditional techniques like PCA for its benefit. As stated in [195, 198], PCA is exploited at its best for feature extraction, selection, and reduction to achieve higher accuracy and performance quality. PCA is one of the best preprocessing methods considered to date for improvised spectral dimension reduction [180], proper selection of spectral bands and their multiscale features in a segmented format [181, 199], noise-reduced spectral analysis [27], and feature extraction [130, 196]. PCA, in collaboration with SVM [195, 200], DL for feature reduction and better classification [182, 183], CNN with multiscale feature extraction [188, 189], and sparse tensor technology [190], has highly been appreciated as soulful research. All these recent time collaborations and a special honor to the merging of ICA-DCT with CNN cited in [191] are the evidence that although PCA is categorized under traditional methods, it is supremely relevant for its significant usefulness in handling HSIs.

Some other hybridizations are also explored by researchers, such as SRC with mathematical index of divergence-correlation [192], Gabor-cube filter [193], and ELM [83, 85]; ELM with CNN [86] and TL [26]; AL based on super-pixel profile [201, 202], AL with CNN [203], CapsNet [204], CNN [204, 205], and TL [151, 184]; CNN with attention-aided methodology [172, 173, 185] and GAN [186]; GAN with dynamic neighborhood majority voting mechanism [194, 197], CapsNet [175, 176, 206, 207]; and TL with MRF [70]. These articles depict the highly tenacious performance with literal mitigation of the computational complexities enforced on the raw HSI data to build a strong and enhanced model for achieving higher accuracy than ever.

*RI 6: What are the latest emerging techniques associated with addressing classifying HSIs?*

Ans: The following are the most recent research studies that have enlightened a new path of dealing with the purpose:

- *DSVM*: The latest and novel concept incorporates DL facilities with traditional kernel SVM. This combines four deep layers of kernels with SVM being the hidden layer units, namely, exponential and gaussian radial basis function (ERBF and GRBF), neural and polynomial [208]. This approach has outperformed several efficient DL methods with nearly 100% accuracy for IP and UP datasets.
- *Conditional Random Fields (CRFs)*: These are the structured generalization of multinomial logistic regression in the form of graphical models based on a priori continuity considering the neighboring pixels of analogous spectral signatures that possess the same labels. They extensively explore the hidden spectral-contextual information. In [146], CRF incorporates with semi-supervised GAN whose trained discriminators produce softmax predictions that are guided by dense CRFs graph constraints to improve HSI classification maps. A collaboration between 3D-CNN and CRF has been proposed in [209] to make a deep CRF capable of extracting the semantic correlations between patches of hypercubes by CNN's unary and pairwise potential functions. A semi-supervised approach is depicted in [210], embedding subspace learning and 3D convolutional autoencoder to remove redundancy in joint features and obtain class sets using an iterative algorithm. In [211], CRF with Gaussian edge potentials associated with deep metric learning (DML) classifies HSI data pixelwise using the geographical distances between pixels and the Euclidean distances between the features. A novel framework using HSI feature learning network (HSINet) with CRF is proposed [212] that is a trainable end-to-end DL model with backpropagation that extracts joint features, edges, and colors based on subpixel, pixel, and super-pixels. In [213], a decision fusion model including CRF and MRF is built based on sparse unmixing and soft classifiers output.
- *Random Forest (RF)*: It is an efficient algorithm that ensembles regression and classification tree. It enables the HSI classification model to be noise-tolerant, inherent in the multiclass division, robustness in parallelism, and speed. In [214], RF is compared to the DL algorithm, which outshined the classification accuracy. A new framework of cascaded RF is shown in [215] that uses the boosting strategy to generate and train base classifiers and Hierarchical Random Subspace Method to select features and suitable base classifiers based on the diversity of the features. A novel collaboration of semi-supervised learning and AL and RF is featured in [216], where the queries based on spatial information are fed to AL, and then, the labeled samples are classified by RF through semi-supervision. [217, 218] depicts a deep cube CNN model that extracts pixelwise joint features and is classified by RF.
- *Graph Convolutional Network (GCN)*: A descendent of CNN, a structure designed to generalize and convert the convolution data to graph data. It consists of three steps feature aggregation, feature transformation, and classification. Being an expert in graphical modeling considers the spatial interrelations between the classes at its best. In [219], the different unique features collected from CNN and GCN are fused additive, elementwise, and concatenated way. A new framework of globally consistent GCN is introduced in [220], which first generates a spatial-spectral local optimized graph whose global high-order neighbors obtain the enriched contextual information employing the graph topological consistent connectivity; at last, those global features determine the classes. [221] shows the concept of a dual GCN network, which works with a limited number of training samples, where first extricates all the significant features and second learns label distribution. A novel idea of deep attention GCN is introduced in [222] based on similarity measurement criteria between the mixed measurement of a kernel-spectral angle mapper and spectral information divergence to accumulate analogous spectra. [223] emerges as a collaboration between CNN and GCN to extract pixel and super-pixelwise joint features by learning small-scale regular regions and large-scale irregular regions.

## 6. Conclusion

This article depicts the various technologies and procedures used for HSI classification since the dawn of its invention to date. There are many barriers to dealing with such high-band data as HSI mentioned above. Despite that, many researchers have taken their interest in this field to improvise the existing techniques or even invent new ones throughout the last decade. As per the considerable improvement in technologies and the introduction of ML into the classification issues of HSI, it has become more accurate than traditional and contemporary state-of-art methodologies. As a result, DL has emerged as the most eminent work tool for HSI classification for the last half of this decade. The more the researchers focused on this, the more they explored the remote sensing and space imagery features.

This review article bears the individual information for every method and their submethods about their performance, research gaps, and achievements. In addition, it appends a novel research methodology that makes this work more distinctive than others. After going through each methodology's minute details, the most significant inferences have been drawn, which add further novelty to our work. Also, it shows a path of choosing an appropriate technique and its alternatives for future researchers, hence alleviating its creativity and uniqueness, above all other contemporary review works on this subject. Also, it provides the details of the most recent research scenario on HSI classification and some of the currently developed techniques that might be acutely useful in several future research. Our study holds the uniqueness and the novelty regarding several aspects, such as the following: (1) it includes the research works carried out in the last decade, that is, 2010–2020, and the most recent papers of the previous year, i.e., 2021, and we have mentioned it in Section 3; (2) the number of papers referred here is above 200, outnumbering other review papers; (3) the review is carried out by selecting the most appropriate papers solely dedicated to our subject of interest, that is, machine learning techniques serving the purpose of hyperspectral image classification. Then, the findings from those works of literature are systematically arranged in the tabular format (Tables 1–12); (4) the objective behind this review work is expressed by RQ 1–6. Also, they provide a clear view of the recent technological advances and applications that the researchers are developing in recent times; (5) Table 14 provides an explicit idea of the pros and cons of each ML technique described in this manuscript when applied for classifying hyperspectral images, which will help the researchers in their future research; and (6) the researcher who wishes to write a literature review can follow our proposed methodology that depicts the flow of work in a methodical way. [224].

## 7. Limitations of Present Work and Its Future Scope

The study has some limitations: (i) we have used fewer keywords in the current research (ii) we only focused on seven popular ML techniques; (iii) we briefly explain the emerging methodologies; and (iv) the experimental details are not fully discussed.

As a future proposition, we would like to explore more keywords, more techniques, and more studies that offer a better understanding of other learning methods, both traditional and contemporary. In addition, there are several instances of hybrid strategies along with some more eminent and latest ML/DL techniques that we shall look forward to exploring in both qualitative and quantitative manner.

## Figures and Tables

**Figure 1:** The statistical pie-charts of screened articles on ML/DL techniques used for HSI classification (source: SCI, SCIE, Scopus, WoS).

**Figure 2:** The statistical bar graph of screened articles on ML/DL techniques used for HSI classification from 2015 to 2021 (source: SCI, SCIE, Scopus, WoS): (a). ML. (b). DL.

**Figure 3:** The categories of the eminent machine learning techniques used for HSI classification.

**Figure 4:** Classification strategy by multiclass SVM.

**Figure 5:** Given the green nodes, the black node is independent of other nodes.

**Figure 6:** Principle of active learning.

**Figure 7:** The network structure of stacked autoencoders; input X-to-E is the encoding phase; E-to-output Y is the decoding phase.

**Figure 8:** The CNN architecture deploying the layers.

**Figure 9:** The RNN structure with recurrent neurons.

**Figure 10:** The detailed DBN structure.

**Figure 11:** The GAN architecture.

**Figure 12:** The principle of transfer learning.

**Table 1:** Summary of review of HSI classification using SVM.

Year	Method used	Dataset and COA	Research remarks and future scope
2011	Multiclass SVM [38]	San Diego3—98.86%	Outperforms traditional SVM and deals better with Hugh's effect
2012	Fuzzy decision tree-support vector machine (FDT-SVM) [39]	Washington DC mall—94.35%	Efficient testing accuracy truncated computational and storage demand, understandable edifices, and reduction of Hugh's effect
2014	Semi-supervised SVM kernel-spectral fuzzy C-means (KSFCM) [40]	IP—98.52%	Enhanced classification and clustering by fully exploring both labeled and unlabeled samples
2014	SVM-radial basis function (SVM-RBF) [41]	IP—88.7%, UP—94.7%	Outperforms other existing kernel-based methods
2015	Regional kernel-based SVM (RKSVM) [42]	UP—95.40%, IP—92.55%	Outperforms pixel-point-based SVM-CK
2017	Multiscale segmentation of super-pixels (MSP-SVMsub) [43]	UP: MSP-SVMsub—97.57%, IP: MSP-SVMsub-95.28%	Solving classic OBIC-based methods with difficulties determining the appropriate segmentation size reduces the Hughes phenomenon
2018	Extended morphological profiles (EMP), differential morphological profiles (DMP), Gabor filtering with SVM [44]	UP: MFSVM-GF—98.46%, IP: MFSVM-GF—98.01%	Outruns several advanced classifiers: SVM, super-pixel-based SVM, SVM-CK, multifeature SVM, EPF
2019	SVM-PCA [24]	IP—91.37%, UP—98.46%	Outperforms Naïve Bayes, decision tree k-NN

**Table 2:** Summary of review of HSI classification using sparse representation.

Year	Method used	Dataset and COA	Research remarks and future scope
2013	Kernel sparse representation classification (KSRC) [45]	IP—96.8%, UP—98.34%, KSC—98.95%	Lacks in devising automatic window size collection of spatial image quality, and filtering degree of class spatial relations

2014	Multiscale adaptive sparse representation (MASR) [46]	UP—98.47%, IP—98.43%, SV—97.33%	MASR outperformed the JSRM single-scale approach and several other classifiers on classification maps and accuracy
			The structural dictionary desired to be more inclusive and trained by discriminative learning algorithms

2015	Sparse multinomial logistic regression (SMLR) [47]	IP—97.71%, UP—98.69%	Being a pixelwise supervised method, its performance is better than other contemporary methods
			The model can be improved via more technical validations, exploitation of MRF, and structured sparsity-inducing norm that enhances the interpretability, stability, and identity of the model learned

2015	Super-pixel-based discriminative sparse model (SBDSM) [377]	IP—97.12%, SV—99.37%, UP—97.33%, Washington DC mall—96.84%	The advantages of this model lie in harnessing spatial contexts effectively through the super-pixel concept, which is better in performance speed and classification accuracy
			Determination of a supplementary and systematic way to adjust the count of super-pixels to various conditions and apply SR to other remote sensing practices

2015	Shape-adaptive joint sparse representation classification (SAJSRC) [48]	IP—98.45%, UP—98.16%, SV—98.53%	Local area shape-adapted for every test pixel rather than a fixed square window for adaptive exploration of spatial PCs, making the method outperforms other corresponding methods
			Region searching based on shape-adaption can be used instead of the reduced dimensional map to reconnoiter complete spatial information of the actual HSI

2017	Multiple-feature-based adaptive sparse representation (MFASR) [49]	IP—97.99%, UP—98.39%, Washington DC mall—97.26%	SA regions' full utilization of all embedded joint features makes the method superior to some cutting-edge approaches
			Enhancement of the proposed method in the future by selecting features automatically and improving dictionary learning to reduce the computational cost

2018	Weighted joint nearest neighbor and joint sparse representation (WJNN-JSR) [50]	UP—97.42%, IP— 93.95%, SV—95.61%, Pavia center—99.27%	The model was improved using the Gaussian weighted method and incorporates the conventional test pixel area to achieve a new measure of classification knowledge: The Euclidean-weighted joint size
			Creating more effective approaches to applying the system and further increasing classification accuracy are taken as future work

2019	Log-Euclidean kernel-based joint sparse representation (LogEKJSR) [51]	IP—97.25%, UP—99.06%, SV—99.36%	Specializes in extracting covariance traits from a spatial square neighborhood to calculate the analogy of matrices with covariances employing the conventional Gaussian form of Kernel
			Creation of adaptive local regions using super-pixel segmentation methods and learning the required kernel using multiple kernel learning methods

2019	Multiscale super-pixels and guided filter (MSS-GF) [52]	IP—97.58%, UP—99.17%	Effective spatial and edge details in his, various regional scales to build MSSs to acquire accurate spatial information, and GF improved the classification maps for near-edge misclassifications
			Additional applications of efficient methods to extract local features and segment super-pixels are added as future work

2019	Joint sparse representation—self-paced learning (JSR-SPL) [53]	IP—96.60%, SV—98.98%	The findings are more precise and reliable than other JSR methods

2019	Maximum-likelihood estimation based JSR (MLEJSR) [54]	IP—96.69%, SV—98.91%, KSC—97.13%	The model is reliable in terms of outliers

2020	Global spatial and local spectral similarity-based manifold learning-group sparse representation-based classifier (GSLS-ML-GSRC) [55]	UP—93.42%, Washington DC mall—91.64%, SV—93.79%	The said fusion makes the method outperform other contemporary methods focused on nonlocal or local similarities

2020	Sparse-adaptive hypergraph discriminant analysis (SAHDA) [56]	Washington DC mall—95.28%	Effectively depict the multiple complicated aspects of the HSI and will be considered for future spatial knowledge

**Table 3:** Summary of review of HSI classification using MRF.

Year	Method used	Dataset and COA	Research remarks and future scope
2011	Adaptive-MRF (a-MRF) [59]	IP—92.55%	Handles homogeneous problem of “salt and pepper” areas and the possibility of overcorrection impact on class boundaries

2014	Hidden MRF and SVM (HMRF-SVM) [60]	IP—90.50%, SV—97.24%	Outperforms SVM and improves overall accuracy outcomes by nearly 8% and 3.2%, respectively

2014	Probabilistic SR with MRF-based multiple linear logistic (PSR-MLL) [61]	IP—97.8%, UP—99.1%, Pavia center—99.4%	Exceeds other modern contemporary methods in terms of accuracy

2014	MRF with Gaussian mixture model (GMM-MRF) [62]	UP(LFDA-GMM-MRF)-90.88% UP(LPNMF-GMM-MRF)—94.96%	Advantageous for a vast range of operating conditions and spatial-spectral information to preserve multimodal statistics
			GMM classificatory distributions are to be considered in the future

2011	MRF with sparse multinomial logistic regression classifier—spatially adaptive total variation regularization (MRF-SMLR-SpATV) [63]	UP—90.01%, IP—97.85%, Pavia center—99.23%	Efficient time complexity of the model
			Improvisation of the model by implementing GPU and learning dictionaries are the future agendas

2016	Multitask joint sparse representation (MJSR) and a stepwise Markov random filed framework (MSMRF) [64]	IP—92.11%, UP—92.52%	The gradual optimization explores the spatial correlation, which significantly improves the effectivity and accuracy of the classification

2016	MRF with hierarchical statistical region merging (HSRM) [65]	SVMMRF-HSRM: IP—93.10%, SV—99.15%, UP— 86.52%; MLRsubMRF-HSRM-IP—82.60%, SV—88.16%, UP—95.52%	Better solution to the technique of majority voting that suffers from the problem of scale choice
			Considering the spatial features in the spatial prior model of objects of the different groups in the future

2018	Integration of optimum dictionary learning with extended hidden Markov random field (ODL-EMHRF) [66]	ODL-EMHRF-ML-IP—98.56%, UP—99.63%; ODL-EMHRF-EM-IP—98.47%, UP—99.58%	The method has been proven to be better than SVM-associated EMRF

2018	Label-dependent spectral mixture model (LSMM) fused with MRF (LSMM-MRF) [67]	The Konka image—94.19%, the shipping scene—66.45%	Efficient unsupervised classification strategy that considers spectral information in mixed pixels and the impact of spatial correlation
			Enhanced theoretical derivations of EM steps

2019	Adaptive interclass-pair penalty and spectral similarity information (aICP2-SSI) along with MRF and SVM [68]	UP—98.10%, SV—96.40%, IP— 96.14%	Outperforms other MRF-based methods
			More efficient edge-preserving strategies, more spectral similitude, and class separable calculation methods as future research

2019	Cascaded version of MRF (CMRF) [69]	IP—98.56%, Botswana—99.32%, KSC—99.24%	Backpropagation tunes the model parameters and least computation expenses

2020	Fusion of transfer learning and MRF (TL-MRF) [70]	IP—93.89%, UP—91.79%	TL is taken to be very effective for HSI classification
			Future research for reducing the number of calculations involved in the existing

2020	MRF with capsule net (caps-MRF) [71]	IP—98.52%, SV—99.74%, Pavia center—99.84%	Ensures that relevant information is preserved, and the spatial constraint of the MRF helps achieve more precise model convergence
			The combination of CapsNet with several postclassification techniques

**Table 4:** Summary of review of HSI classification using ELM.

Year	Method used	Dataset and COA	Research remarks and future scope
2014	Ensemble extreme learning machines (E^2^LM)-bagging-based ELMs (BagELMs) and AdaBoost-based (BoostELMs) [72]	UP—94.3%, KSC—97.71%, SV—97.19%	BoostELM performs better than kernel and other EL methods
			Performance of other differential or nondifferentiable activation functions

2015	Kernel-based ELM—composite kernel (KELM-CK) [75]	IP—95.9%, UP—93.5%, SV—96.4%	Outperforms other SVM-CK-based models

2015	ELM's two-level fusions: feature-level fusion (FF-ELM) and mixing ELM classifier two levels of fusions: feature-level fusion (FF-ELM) [76]	FF-ELM: UP—98.11%, IP—92.93%, SV—99.12%; DF-ELM—UP—99.25%, IP—93.58%, SV—99.63%	Outperforms basic ELM models

2016	Hierarchical local-receptive-field-based ELM (HL-ELM) [77]	IP—98.36%, UP—98.59%	Surpasses other ELM methods in terms of accuracy and training speed

2017	Genetic-firefly algorithm with ELM (3FA-ELM) [78]	HyDice DC mall—97.36%, HyMap—95.58%	Low complexity (ELM), better adaptability, and searching capability (FA)
			Execution time needs to be reduced in future

2017	Local receptive fields-based kernel ELM (LRF-KELM) [79]	IP—98.29%	Outperforms other ELM models

2017	Distributed KELM based on MapReduce framework with Gabor filtering (DK-Gabor-ELMM) [80]	IP—92.8%, UP—98.8%	Outperforms other ELM models

2017	Loopy belief propagation with ELM (ELM-LBP) [81]	IP—97.29%	Efficient time complexity

2018	Mean filtering with RBF-based KELM (MF-KELM) [82]	IP—98.52%	The model offers the most negligible computational hazard

2018	Augmented sparse multinomial logistic ELM (ASMLELM) [83]	IP—98.85%, UP—99.71%, SV—98.92%	Improved classification accuracy by extended multi-attribute profiles and more SR

2018	ELM with enhanced composite feature (ELM-ECF) [84]	IP—98.8%, UP—99.7%, SV—99.5%	Low complexity and multiscale spatial feature for better accuracy
			Incorporate feature-fusion technology

2019	Local block multilayer sparse ELM (LBMSELM) [85]	IP—89.31%, UP—89.47%, SV—90.03%	Performs anomaly and target detection. Reduced computational overhead and increased classification accuracy by inverse free; saliency detection and gravitational search

2019	ELM-based heterogeneous domain adaptation (EHDA) [25]	HU-DC —97.51%, UP-DC —96.63%, UP-HU —97.53%	Outperforms other HDA methods. Invariant feature selection

2019	Spectral-spatial domain-specific convolutional deep ELM (S^2^CDELM) [86]	IP—97.42%, UP—99.72%	Easy construction with high training-testing speed
			Merge of DL with ELM
2020	Cumulative variation weights and comprehensive evaluated ELM (CVW-CEELM) [87]	IP—98.5%, UP—99.4%	Accuracy achieved due to the weight determination of multiple weak classifiers. Multiscale neighborhood choice and optimized feature selection

**Table 5:** Summary of review of HSI classification using active learning.

Year	Method used	Dataset and COA	Research remarks and future scope
2008	AL with expectation-maximization-binary hierarchical classifier (BHC-EM-AL) and maximum-likelihood (ML-EM-AL) [90]	Range: KSC-90-96%, Botswana—94-98%	Better learning levels than the random choice of data points and an entropy-based AL
			Measurement of the efficacy of the active learning-based knowledge transfer approach while systematically increasing the spatial/temporal segregation of the data sources

2010	Semi-supervised-segmentation with AL and multinomial logistic regression (MLR-AL) [91]	IP—79.90%, SV—97.47%	Innovative mechanisms for selecting unlabeled training samples automatically, AL to enhance segmentation results
			Testing the segmentation in various scenarios influenced by limited a priori accessibility of training images

2013	Maximizer of the posterior marginal by loopy belief propagation with AL (MPM-LBP-AL) [92]	IP—94.76%, UP—85.78%	Improved accuracy than previous AL applications
			Use parallel-computer-architectures such as commodity—clusters or GPUs to build computationally proficient implementation

2015	Hybrid AL-MRF, that is, uncertainly sampling breaking ties (MRF-AL-BT), passive selection approach random sampling (MRF-AL-RS), and the combination (MRF-AL-BT + RS) [93]	IP—94.76%, UP—85.78% (MRF-AL-RS provides the highest accuracies)	Outperforms conventional AL and SVM AL methods due to MRF regularization and pixelwise output
			Merge the model with other effective AL methods and test them with a limited number of training samples

2015	Integration of AL and Gaussian process classifier (GP-AL) [94]	IP—89.49%, Pavia center—98.22%	Empirical autonomation of AL achieves reasonable accuracy
			Adding diversity criterion to the heuristics and contextual information with the model and reducing computation time

2016	AL with hierarchical segmentation (HSeg) tree: adding features and adding samples (Adseg_AddFeat + AddSamp) [95]	IP—82.77%, UP—92.23%	Outruns several baseline methods-selecting appropriate training data from already existing labeled datasets and potentially decreasing manual laboratory labeling
			Reduce the computational time that limits its applicability on large-scale datasets

2016	Multiview 3D redundant discrete wavelet transform-based AL (3D-RDWT-MV-AL) [96]	HU—99%, KSC—99.8%, UP—95%, IP—90%	The precious method as a combination of an initial process with AL, improved classification

2017	Discovering representativeness and discriminativeness by semi-supervised active learning (DRDbSSAL) [97]	Botswana—97.03%, KSC—93.47%, UP—93.03%, IP—88.03%	Novel approach with efficient accuracy

2017	Multicriteria AL [98]	KSC—99.71%, UP—99.66%, IP—99.44%	Surpasses other existing AL methods regarding stability, accuracy, robustness, and computational hazard
			A multi-objective optimization strategy and the usage of advanced attribute-based profile features

2018	Feature-driven AL associated with morphological profiles and Gabor filter [99]	IP—99.5%, UP—99.84%, KSC—99.53% (Gabor-BT)	A discriminative feature space is designed to gather helpful information into restricted samples

2018	Multiview intensity-based AL (MVAL)-multiview intensity-based query-representative strategy (MVIQ-R) [100]	UP—98%, Botswana—99.5%, KSC—99.9%, IP—95%	Focus on pixel intensity obtains unique feature and hence better performance
			Selection of combination of optimal attribute features

2019	Super-pixel with density peak augmentation (DPA)-based semi-supervised AL (SDP-SSAL) [101]	IP—90.08%, UP—85.61%	Novel approach proposed based on super-pixels density metric
			Development of a pixelwise solution to produce super-pixel-based neighborhoods

2020	Adaptive multiview ensemble spectral classifier and hierarchical segmentation (Ad-MVEnC_Spec + Hseg) [102]	KSC—97.63%, IP—87.1%, HU—93.3%	Enhancement in the view sufficiency, and promotion of the disagreement level by the dynamic view, provides lower computational complexity due to parallel computing

2020	Spectral-spatial feature fusion using spatial coordinates-based AL (SSFFSC-AL) [103]	IP—100%, UP—98.43%	High running speed can successfully address the “salt and pepper” phenomenon but drops a few if similar class samples are distributed in different regions differently
			The sampling weight parameter conversion to an adaptive parameter is adjusted adaptively as the training samples are modified

**Table 6:** Summary of the review of HSI classification using deep learning—AE.

Year	Method used	Dataset and COA	Research remarks and future scope
2013	Autoencoders (AE) [110]	Error rate: KSC—4%, Pavia city—14.36%	This article opened a considerable doorway of research, including other deep models for better accuracy

2014	Stacked autoencoder and logistic regression (SAE-LR) [113]	KSC—98.76%, Pavia city—98.52%	Highly accurate in comparison to RBF-SVM and performs testing in optimized time limit than SVM or KNN but fails in training time efficiency

2016	Spatial updated deep AE with collaborative representation-based classifier (SDAE-CR) [114]	IP—99.22%, Pavia center—99.9%, Botswana—99.88%	Highly structured in extracting high specialty deep features and not the hand-crafted ones and accurate
			Improving the deep network architecture and selection of parameters

2019	Compact and discriminative stacked autoencoder (CDSAE) [115]	UP—97.59%, IP—95.81%, SV—96.07%	Efficient in dealing with feature space in low dimension, but the computation cost is high as per architecture size

2021	Stacked autoencoder with distance-based spatial-spectral vector [116]	SV—97.93%, UP—99.34%, surrey—94.31%	Augmentation of EMAP features with the geometrically allocated spatial-spectral feature vectors achieves excellent results. Better tuning of hyperparameter and more powerful computational tool required
			Improving the training model to become unified and classified in a more generalized and accurate way

**Table 7:** Comparison of convolutional layers.

Arguments	Convolution layer	Pooling layer	Fully connected layer
Input	(i) 3D-cube, preceding set of feature maps	(i) 3D-cube, preceding set of feature maps	(i) Flattened-3d-cube, preceding set of feature maps

Parameters	(i) Kernel counts	(i) Stride	(i) Number of nodes
	(ii) Kernel size	(ii) Size of window	(ii) Activation function: selected based on the role of the layer. For aggregating info-ReLU. For producing final classification—softmax
	(iii) Activation function (ReLU)		
	(iv) Stride		
	(v) Padding		
	(vi) Type and value of regularization		

Action	(i) Application of filters made of small kernels to extricate features	(i) Reduction of dimensionality	(i) Aggregate information from final feature maps
	(ii) Learning	(ii) Extraction of the maximum of a region average	(ii) Generate final classification
	(iii) One bias per filter	(iii) Sliding window framework	
	(iv) Application of activation function on each feature map value		

Output	(i) 3D-cube, a 2D-map per filter	(i) 3D-cube, a 2D-map per filter, reduced spatial dimensions	(i) 3D-cube, a 2D-map per filter

**Table 8:** Summary of review of HSI classification using deep learning—CNN.

Year	Method used	Dataset and COA	Research remarks and future scope
2015	Convolutional neural network and multilayer perceptron (CNN-MLP) [120]	Pavia city—99.91%, UP—99.62%, SV—99.53%, IP—98.88%	Far better than SVM, RBF mixed classifiers, the effective convergence rate can be useful for large datasets
			Detection of human behavior from hyperspectral video sequences

2016	3D-CNN [121]	IP—98.53%, UP—99.66%, KSC—97.07%	A landmark in terms of quality and overall performance
			Mapping performance to be accelerated by postclassification processing

2016	Spectral-spatial feature-based classification (SSFC) [122]	Pavia center—99.87%, UP—96.98%	Highly accurate than other methods
			Inclusion of optimal observation scale for improved outcome

2016	CNN-based simple linear iterative clustering (SLIC-CNN) [123]	KSC—100%, UP—99.64, IP—97.24%	Deals with a limited dataset use spectral and local-spatial probabilities as an enhanced estimate in the Bayesian inference

2017	Pixel-pair feature enhanced deep CNN (CNN-PPF) [124]	IP—94.34%, SV—94.8%, UP—96.48%	Overcomes the significant parameter and bulk-data problems of DL, PPFs make the system unique and reliable, and voting strategy makes the more enhanced evaluations in classification

2017	Multiscale 3D deep convolutional neural network (M3D-DCNN) [125]	IP—97.61%, UP—98.49%, SV—97.24%	Outperforms popular methods like RBF-SVM and combinations of CNNs
			Removing data limitations and improving the network architecture

2018	2D-CNN, 3D-CNN, recurrent 2D-CNN (R-2D-CNN), and recurrent 3-D-CNN (R-3D-CNN) [126]	IP-99.5%, UP—99.97%, Botswana—99.38%, PaviaC—96.79%, SV—99.8%, KSC—99.85%	R-3D-CNN outperforms all other CNNs mentioned and proves to be very potent in both fast convergence and feature extraction but suffers from the limited sample problem
			Applying prior knowledge and transfer learning

2019	3D lightweight convolutional neural network (CNN) (3D-LWNet) [127]	UP—99.4%, IP—98.87%, KSC—98.22%	Provides irrelevance to the sources of data
			Architecture is to be improvised by intelligent algorithms

2020	Hybrid spectral CNN (HybridSN) [128]	IP—99.75%, UP—99.98%, SV—100%	Removes the shortfalls of passing over the essential spectral bands and complex, the tedious structure of 2D-CNN and 3D-CNN exclusively and outruns all other contemporary CNN methods superiorly, like SSRN and M-3D-CNN

2020	Heterogeneous TL based on CNN with attention mechanism (HT-CNN-attention) [129]	SV—99%, UP—97.78%, KSC—99.56%, IP—96.99%	Efficient approach regardless of the sample selection strategies chosen

2020	Quantum genetic-optimized SR based CNN (QGASR-CNN) [27]	UP—91.6%, IP—94.1%	With enhanced accuracy, overfitting and “salt-and-pepper” noise are resolved
			Improvement of operational performance by the relation between feature mapping and selection of parameters

2020	Rotation-equivariant CNN2D (reCNN2D) [130]	IP—97.78%, UP—98.89, SV—98.18%	Provides robustness and optimal generalization and accuracy without any data augmentation

2020	Spectral-spatial dense connectivity-attention 3D-CNN (SSDANet) [131]	UP—99.97%, IP— 99.29%	Higher accuracy but high computational hazard
			Optimization by using other efficient algorithms

**Table 9:** Summary of review of HSI classification using deep learning—RNN.

Year	Method used	Dataset and COA	Research remarks and future scope
2017	Gated recurrent unit-based RNN with parametric rectified tanh as activation function (RNN-GRU-pretanh) [132]	UP—88.85%, HU—89.85%, IP—88.63%	An enhanced model that utilizes the intrinsic feature provided by HS pixels with better accuracy than SVM
			The study is limited to only spectral features
			Incorporation of deep end-to-end convolutional RNN with both spatial-spectral features

2019	Spectral-spatial cascaded recurrent neural network (SSCasRNN) [135]	IP—91.79%, UP—90.30%	Outruns pure RNN and CNN models due to the perfect placement of convolutional and recurrent layers to explore joint information

2020	Geometry-aware deep RNN (Geo-DRNN) [136]	UP—98.05%, IP—97.77%	Due to encoding the complex geometrical structures, the data lack space
			Minimization of memory-occupation

2021	2D and 3D spatial attention-driven recurrent feedback convolutional neural network (SARFNN) [28]	IP—99.15%, HU—86.05%	Integrating attention and feedback mechanism with recurrent nets in two layers, 2D and 3D, enables efficient accuracy

**Table 10:** Summary of review of HSI classification using deep learning—DBN.

Year	Method used	Dataset and COA	Research remarks
2015	Deep belief network and logistic regression (DBN-LR) [137]	IP—95.95%, Pavia City—99.05%	The drawback in training time complexity, it is super-fast testing, and result generating capability outperforms RBF-SVM with EMP

2019	Spectral-adaptive segmented deep belief network (SAS-DBN) [138]	UP—93.15%, HU—98.35%	Capable of addressing the complexities and other subsidiaries of limited samples

2020	Conjugate gradient update-based DBN (CGDBN) [139]	UP—97.31%	Better approach towards stability and convergence of the training model
			High time complexity

**Table 11:** Summary of review of HSI classification using deep learning—GAN.

Year	Method used	Dataset and COA	Research remarks and future scope
2018	Hyperspectral 1D generative adversarial networks (HSGAN) [140]	IP—83.53%	Outperforms CNN, KNN, etc.

2018	3D augmented GAN [143]	SV—93.67%, IP—91.1%, KSC—98.12%	Data augmentation solved the problem of overfitting and improved class accuracy

2019	Conditional GAN with conditional variational AE (CGAN-CVAE) [144]	UP—83.85%, DC Mall—89.36%	Semi-supervised and ensemble prediction technique ensures the model's training under limited sample conditions

2020	Semi-supervised variational GAN (SSVGAN) [145]	UP—84.35%, Pavia Center—97.15%, DC Mall—92.21%, Jiamusi—64.76%	Outperforms other GAN variants, that is, CVAEGAN and ACGAN, but it suffers from feature matching, overfitting, and convergence problem
			Correction through metric learning method

2020	Spectral-spatial GAN-conditional random field (SS-GANCRF) [146]	IP—96.3%, UP—99.31%	Enhanced classification capability
			Creating an end-to-end training system, graph constraint placed on the convolutional layers

2021	Adaptive weighting feature-fusion generative adversarial network (AWF^2^-GAN) [147]	IP—97.53%, UP—98.68%	Exploration of the entire joint feature space and fusion of them, joint loss function, and the central loss gained intraclass sensitivity from local neighboring areas and offered an efficient spatial regularization outcome

2021	Variational generative adversarial network with crossed spatial and spectral interactions (CSSVGAN) [148]	IP—93.61%, UP—99.11%, SV—97%	Increased classification potential by utilizing transformer and GAN

**Table 12:** Summary of review of HSI classification using transfer learning.

Year	Method used	Dataset and COA	Research remarks and future scope
2018	Deep mapping-based heterogeneous transfer learning model (DLTM) [150]	Washington DC Mall—96.25%	Capable of binary classification
			Improvisation to multiclass classification

2018	AL with stacked sparse autoencoder (AL-SSAE) [151]	UP—99.48%, center of Pavia—99.8%, SV— 99.45%	Domains, both source, and target possess finely tuned hyperparameters
			Architectural parameters need to be modified further to enhance the classification accuracy

2020	Heterogeneous TL based on CNN with attention mechanism (HT-CNN-attention) [152]	SV—99%, UP—97.78%, KSC—99.56%, IP—96.99%	Efficient approach regardless of the sample selection strategies chosen

2020	ELM-based ensemble transfer learning (TL-ELM) [26]	UP—98.12%, Pavia center—96.25%	Efficient accuracy and transferability with high training speed
			Inclusion of SuperPCA and knowledge transfer

2020	Lightweight shuffled group convolutional neural network (abbreviated as SG-CNN) [153]	Botswana—99.67%, HU—99.4%, Washington DC—97.06%	Fine-tuned model as compared to CNN architectures, low computational cost for training
			Inclusion of more grouped convolutional architectures

2021	Super-pixel pooling convolutional neural network with transfer learning (SP-CNN) [154]	SV—95.99%, UP—93.18%, IP—94.45%	More excellent parameter optimization with more accuracy using a limited number of samples and in a very short period for both training and testing
			Optimal super-pixel segmentation and merging with different CNN architectures

**Table 13:** Comparison between ML and non-ML techniques for HSI classification.

Methods	Advantages	Disadvantages
Classical state-of-art techniques	(i) Simple structure and design	(i) High space complexity due to the storage of bulk data
	(ii) Less time consumption	(ii) Based on empirical identities, hence a tedious workpiece
	(iii) Easy to implement	(iii) Feature selection and extraction are not accurate
	(iv) Dimension handling skillfully by PCA and ICA	(iv) Suffers from limited labeled sample problem, Hughes phenomenon, and noise
	(v) Better binary and moderate multiclass classification by kernel and SVM	

Advanced machine learning techniques	(i) Easy dealing with high-dimensional data, that is, troubles of Hughes phenomenon removed	(i) The construction of the model is difficult due to its complex network-alike structure
	(ii) Equally manipulative to labeled and unlabeled samples	(ii) High time complexity due to training and testing of the huge amount of raw HSI data
	(iii) Precise and meticulous choice of features	(iii) Extremely expensive design
	(iv) High-end-precise models to deal with real hypercubes, hence, top-notch classification accuracy	(iv) Strenuous to implement
	(v) Removes overfitting, noises, and other hurdles to a much greater extent	
	(vi) Mimics the human brain to solve multiclass problems	

**Table 14:** The advantages and challenges of the ML- and DL-based techniques for HSI classification.

ML/DL techniques	Advantages	Challenges
Support vector machine	(i) Robust in terms of outliers, Hughes effect, and dimensions as its reduction is not primarily necessary [32, 41, 43]	(i) It works very well for binary classification but fails for generating accurate classes for multiclass problems [31]
	(ii) Supports both supervised, semi-supervised, and unsupervised problems with less overfitting risks [24, 33, 37, 44]	(ii) Training time is high for high-class datasets like HSI [31, 32]
	(iii) Form of a sigmoid kernel that deals better than the rest of the previous for unlabeled and unstructured HSI datasets [35, 40–42]	(iii) Difficulty in fine-tuning the parameters [41, 42]
	(iv) The capability of solving the classification problem for both binary and multiclass problems by outperforming several methods [39]	(iv) Complex interpretability [33, 35]
	(v) Can improve the performance if assisted with other supporting methods [36, 40–42]	(v) Lack of easy generalization to the datasets having multiple classes [33, 35]
		(vi) Complexity in building the model due to a lack of sufficient labeled samples [31, 32]

Sparse representation and classification	(i) A dictionary with relevant data is used for learning with a minimal number of optimal parameters [45, 46]	(i) Making the dictionary considers high expense overheads [50]
	(ii) Builds precise and powerful classification models with higher interpretability through sparse coding [49, 50, 54]	(ii) The dictionary or the coding might cause loss of information [48, 178]
	(iii) Proper memory usage in an optimized manner [53, 55, 178]	(iii) Difficulties in representing such high-profile with higher resolution image data like HSI through the sparse matrix [47, 48]
	(iv) Reduces the estimated variance between the classes to produce better outcomes [49, 56, 178]	

Markov random field	(i) Works well for a wide range of unstructured problems and no direct dependency between classes and the parameters [67, 69]	(i) Normalization of data might be hectic for high dimension data [63, 70]
	(ii) Better denoising effect [59]	(ii) Suffers from the lack of training undirected data that might not be possible to represent graphically [61, 62]
	(iii) Robust for both spatial and spectral distributions [62, 64]	(iii) Poor interpretability [63, 68]
	(iv) Time complexity is low due to the graphical representation of data [63]	

Extreme learning machines	(i) Less training time and faster learning rate as compared to previous methods [86]	(i) Higher computational hazard [76–80]
	(ii) Avoidance for local minima and finishes job in single iteration [83, 87]	(ii) The wrong choice of an optimal amount of the hidden layer neurons may cause redundancy in the model and hence affect the classification accuracy [85, 86]
	(iii) Advantageous for overfitting caused due to several bands in HSIs [83]	(iii) There is plenty of room for advancements in the algorithm to accommodate itself to be compatible for dealing with HSI data [78, 82, 86]
	(iv) Builds an enhanced model with better prediction performance at the optimized expense [86]	
	(v) Improved generalization ability, robustness, and controllability [78, 84, 85]	

Active learning	(i) A very efficient way of learning for both supervised and semi-supervised problems [91, 97, 101, 103]	(i) Higher computational hazard [76–80]
	(ii) Ease in segregating the interclass and intraclass features through active query sets [91, 95, 102, 103]	(ii) The wrong choice of an optimal amount of the hidden layer neurons may cause redundancy in the model and hence affect the classification accuracy [85, 86]
	(iii) Training speed is comparatively high for not so large-scale data [103]	(iii) There is plenty of room for advancements in the algorithm to accommodate itself to be compatible for dealing with HSI data [78, 82, 86]
	(iv) Knowledge-based solid models can be generated [103]	
	(v) Achieves greater classification accuracies for unlabeled HSIs [95, 102]	

Deep learning	(i) Diverse, unstructured, and unlabeled raw HSI datasets are finely processed where preprocessing of the data is not needed [110, 122, 125, 144]	(i) Suffers from a lack of a large amount of HSI data, which is practically unavailable [123, 136]
	(ii) Possesses the capability to address supervised, semi-supervised, and specifically unsupervised learning problems [127, 128, 137]	(ii) The extreme expense to generate an appropriate model by training a complex data structure like HSIs [114, 139, 148]
	(iii) Expertise in dimension reduction, denoising, feature extraction as embedded properties [27, 114, 124]	(iii) Low interpretability [131, 147]
	(iv) Address in an illustrious manner to the issues such as Hughes phenomenon, overfitting, and convergence. [120, 124, 145]	(iv) Theoretically not sound, hence incomprehensible where an error occurs and its rectification [122, 124, 145]
	(v) Robust and adaptive to new features introduced in the dataset [26, 123, 145]	(v) High time and space complexity and computational hazard [131, 136, 148]
	(vi) The hidden layer neurons are proven to be eminent in training the desired model with a highly qualified prior knowledge (DBN, RNN, CNN) [127, 129, 135, 138]	
	(vii) Computational efficiency with high-performance speed (CNN, SAE) [114, 115, 127, 128]	
	(viii) Data augmentation facility (GAN) [143, 145]	

Transfer learning	(i) Works as a combination of different models, be it traditional or latest machine-lefted techniques, that together brings out a highly improved hybrid model [151, 152]	(i) Data overfitting [150]
	(ii) Capable of transferring knowledge from the source domain, that is , a pretrained model to the target domain, that is, a new model to make it more enriched [151, 152]	(ii) Complex structure of the model [150, 151]
	(iii) Greater feature extraction and selection capability [152]	(iii) Less interpretability
	(iv) Stable model with highly optimized parameters and hyperparameters [154]	(iv) Difficulty in implementation
	(v) High training speed and accuracy with low computational cost [26, 153]	
	(vi) Reduced computational cost and training time complexity [153, 154]	

## Data Availability

Publicly available data are used in this study.

## Acronym

HS: Hyperspectral
HSI: Hyperspectral image
GIS: Geographic Information System
PCA: Principal component analysis
ICA: Independent component analysis
SVM: Support vector machine
SR: Sparse representation
SRC: Sparse representation and classification
MRF: Markov random field
HMRF: Hidden Markov random field
ELM: Extreme learning machine
AL: Active learning
HU: University of Houston
TL: Transfer learning
DL: Deep learning
AE: Autoencoders
SAE: Stacked autoencoders
CNN: Convolutional neural network
RNN: Recurrent neural network
DBN: Deep belief network
GAN: Generative adversarial network
IP: Indian pines
KSC: Kennedy space center
SV: Salinas valley
UP: University of Pavia.
